This article has been retracted.

# Application of Mathematical Models in Economic Variable Input and Output Models under the Scientific Visualization

**DOI:** 10.1155/2022/6269358

**Published:** 2022-02-21

**Authors:** Kai Zheng, Yisheng Liu

**Affiliations:** ^1^Research Institute for the Development of Private Economy, A New Type of Think Tank with Characteristics in Colleges and Universities in Fujian Province, Fujian, Quanzhou, China; ^2^College of International Finance and Trade, Zhejiang Yuexiu University of Foreign Languages, Shaoxing, Zhejiang, China; ^3^School of Political and Social Development, Quanzhou Normal University, Quanzhou, Fujian, China

## Abstract

At present, with the development of society and economy, some new problems have emerged continuously. Among them, the more serious problem is that enterprises pay too much attention to economic benefits, which leads to problems in the development of many enterprises. Therefore, the problem caused by too much emphasis on economic benefits is one of the major economic problems. After this problem, our country's economy began to focus on economic input and output in the subsequent development process. And, related personnel have also studied the economic input-output technology and model, which is an economic quantitative analysis method that has been widely used in various aspects of the economic field since its emergence. This paper firstly elaborates the theoretical knowledge involved, such as economic data, economic variables, and visualization techniques. Secondly it analyzes the application of scientific visualization techniques in the processing of economic variable data, which includes the techniques of preprocessing, mapping, drawing, and displaying the data. Finally, this paper investigates the application of mathematical models in economic variables input and output and the application of mathematical models in economic research, which can help us to better understand and use the knowledge of economics, thus providing strong support for solving practical problems. Also, this helps people to understand and grasp more about the macroarea, microaspect, and even the country as a whole.

## 1. Introduction

Beginning in the late 1970s, some foreign researchers have made in-depth discussions on visualization-related issues, such as measurement, mathematical models, and so on. Since 1980, our country began to pay attention to the fields of scientific visualization theories and methods. In addition, many countries have done a lot of research on the economic input-output model, which makes the economic input-output model more widely used in the economic development of enterprises [1]. The input-output model is mainly used for the analysis of the chain impact of product price changes, the analysis of investment-induced effects, and the analysis of industrial structure adjustment. At present, domestic scholars have not formed a systematic and effective framework to serve quantitative analysis. It is also an important problem to be solved at present to conduct a deeper research on how to establish the relationship between the input and output of a set of economic variables [2].

In summary, this paper mainly studies the following contents:

Mathematics is a highly abstract discipline that covers many fields and has a wide range of applications in economics, sociology, and psychology, among others. We can see that classifying variables from different perspectives often requires the consideration of several factors at the same time. For example, when people are faced with a problem in their lives, they choose to think about all the possible solutions to the problem before making a decision [3]. Mathematical visualization is the use of computer technology to visualize areas that do not require precise data, such as functions and probabilities. It allows us to use existing knowledge to solve practical problems more easily, quickly, and effectively. The variables involved in this process can also produce a certain degree of “backward” effect or partially offsetting effect (which is unpredictability and nonordered error) with time change, thus affecting the effect of mathematical modeling, which makes the visualization theory more comprehensive and accurate to play its proper value [4, 5]. In this paper, we introduce some visualization variables based on previous research and then build a mathematical model and dig deeper into it.

Economic variables are important factors in explaining the production function and can generally be reflected by the ratio of a given output to income. In real life, there are usually one or more economic variables that are related to output, have some correlation, and can be expressed in different quantities. For example: when unit output value = GDP*∗*(*X*1 + *Y*0)/*y*, the sales price of its product is zero; for the same linear equation, it is output per unit × *x* value. That is, each production function has more than two given quantities and another known variable, and each output value has more than two known quantities and another unknown variable [6].

 Mathematical models can concretize abstract, nonquantitative problems, and in practical applications it has a profound impact on people's lives. In the traditional method, some situations are unpredictable or difficult to explain by decision makers, and this method can be used to solve them. The word “precision” first appeared in the mid-19th century. With the progress of the times and the technological revolution, the word “precision” was introduced. A mathematical model is a tool for describing, reasoning, and calculating the relationships between things and the laws arising from changes in their nature by using certain quantitative and quantifiable objects. Precise mathematical models play an important role in economic research, which can help people to simplify complex problems and solve practical problems, so it is getting more and more attention and application [7, 8].

The application of mathematical models is mainly to solve the visualization of economic variables, and in reality, some data cannot be directly obtained, so it needs to be transformed into something that can visually reflect the essential characteristics and inner laws of things, reflect the nature of the problem, or describe things, and other functions are clearer and easier to understand and grasp the interconnection and influence relationship between the phenomena under study. This requires us to pay attention to the actual situation as well as to grasp the development trend of scientific knowledge itself. Mathematical models as an effective method can be used to solve some difficult problems in the visualization of economic variables, which are widely used in many fields [9].

Scientific visualization refers to the realization of human-computer interaction with the knowledge and information involved in the process of data acquisition, processing, and analysis through computer technology, so that people can understand and use it. Essentially, it is a way of thinking. In traditional mathematical models, only the relationship between variables and the internal structure characteristics of variables are usually studied to describe the degree of influence of random events, which ignores its internal laws and state change trends. However, modern visualization can help researchers to understand and analyze the problems, causes, and development prospects in complex systems more deeply, so visualization technology is more and more widely used in mathematical research [10, 11].

The economic data is the basis for the construction of the visualization model. In the process of building it, it is necessary to classify the variables under study and then analyze the interrelationships and internal logical relations between these indicators. For example, for the attribute of production (output), cost of production, etc., it is a function, while for the attribute of consumer demand it is utility. These two sets of regression coefficients and test results are used to determine the level of economic development, how it determines the amount of input, and whether it grows and thus affects the rationality of the visualization modeling, which provide valid support for policy makers.

For mathematical visualization, scholars at home and abroad have carried out research from different angles and achieved some good results. These theories can be used to solve practical problems. There are many related discussions on science abroad. For example, two of the famous foreign economists Kahneman and Delphi put forward the “strategic” concept (Non-Levin); Professor James Gist of Harvard University in the United States believes that visualization is not only an information processing technology or tool, but also a source of human wisdom. The research on mathematical visualization in our country started late, and the research on visualization mainly focuses on economic variables, explanatory variables, and application fields. There is no complete system about how to apply the mathematical model to practice.

Scientific visualization refers to people's intuitive, concrete, and vivid definition of complex problems or phenomena and makes them a clear and easy-to-understand expression through visual and auditory methods. It mainly includes three aspects: the first is to make an accurate judgment on the existence of a large number of uncertain factors in the objective world; the second is to make an abstract generalization of the natural system in essence; the third is to describe the nature and various phenomena involved in the process of social development and their interrelations and interactions. The research model based on visual analysis is shown in Figure 1.

Based on the economic study of scientific visualization, we analyze the following aspects. Firstly, mathematical modeling: In the traditional field of economics, it is usually assumed that a variable can be expressed by a simple formula; secondly, the mathematical methods are improved and refined and applied to real life, converting the data that were impossible or partially unavailable to the results that can be obtained by simply calculating a functional expression, which is called a visualization algorithm. Finally, computer-aided technology is used to combine economic indicators with other nonquantitative factors to obtain quantitative indicators [12].

## 2. Materials and Methods

### 2.1. Data Preprocessing

For data processing we usually use some mathematical methods, such as statistical models, image models, and so on. However, these common econometric research tools often require a large number of complex and detailed models of the sample in practice. Therefore, in this paper, we will select appropriate and reasonable information that can reflect the real situation and representative information as the essence, so as to better provide more useful information for decision makers to make accurate choices and reference data for decision making; at the same time, it can also provide more useful information for specific decision makers, so that they can make more accurate and rational choices. The block diagram of data preprocessing is shown in Figure 2.

In this paper, mathematical tools based on the “least squares” algorithm (SURF) and the LM heuristic algorithm are used to complete the data preprocessing process. Among them, the “least squares” algorithm (SURF) is mainly used for data correction; i.e., when there is only random error in the variables, as described in formula (1), and when there is significant error in the variables, the algorithm is described in formula (2).

(1) $$\begin{array}{c} x^{m}=x+\varepsilon . \end{array}$$

(2) $$\begin{array}{c} x^{m}=x+\varepsilon +b. \end{array}$$

One of the characteristics of display technology is the display of the amount of data that needs to be processed, especially image data. As the resolution of image capture tools increases, the amount of image data per frame increases exponentially. Therefore, the storage and transmission of data have a negative impact, which means that the capacity of internal/external memory must be expanded to increase the speed of data communication. One of the technical methods to overcome this difficulty is to use data compression technology. Traditionally, data compression technology has always been one of the main research materials in digital image processing. Data compression technology can be divided into lossless compression and lossy compression according to the degree of distortion of information after compression. And its compression time is relatively long, but when the data block is processed and compressed, it is prone to overflow. The development of scientific computing screen technology and the development of multimedia computing technology have promoted the development of data compression technology. The current data compression technology can reduce the data storage capacity, but its computational complexity is high, and it needs continuous improvement. In recent years, data compression algorithms and standardization have developed rapidly, and integrated circuits and dedicated hardware used for compression applications have become the main topics of current research. The data compression technology flowchart is shown in Figure 3. The implementation of the data algorithm is in Algorithm 1.

Through this article, we can understand that data compression technology can effectively expand storage capacity and accelerate the speed of data communication; now there are various data compression systems on the market. The performance metrics should include (1) minimum error density; (2) maximum variance rate as well as minimum entropy value; (3) minimum generative model; 4–6 are the missing values of metrics; i.e., the weights and maximum entropy values are selected as the measurement factors without considering the nonordered visualization.

Data compression techniques can be divided into lossless compression and lossy compression according to the degree of distortion to the information after compression. Lossless compression technique is to segment data points with certain characteristics, which is characterized by reducing the amount of information required in random measurements; it is a probability density estimation technique; this can simplify the calculation of statistics. Lossy compression is characterized by a higher compression ratio than lossless compression, but it usually causes distortion after decompression. Also, the number of variables is uncertain and the variables are closely related to each other.

According to the output distribution characteristics of the compressed information source, data compression can be divided into statistical coding and dictionary coding. Statistical compression is one of the earliest compression techniques used and it is associated with classical data compression. Vocabulary encoding is also called LZ encoding. The basic principle is to select a character string from the source output data, save each character string code as an identifier, and use the dictionary search principle to encode the compressed character string and perform character string encoding.

Data compression technology can reduce data storage capacity. The principle of data compression technology is as follows: due to some redundancy between image data, this makes data compression possible. Shannon, the founder of information theory, proposed to treat data as a combination of information and redundancy. The so-called redundancy is due to the high correlation between the pixels of the image, so many coding methods can be used to remove them, so there is no need to reduce the compressed data.

One of the characteristics of visualization technology is the display of the amount of data that needs to be processed. The application of visualization technology in mathematics is mainly reflected in, first, the integration of data and information, through the transformation of complex abstract problems into simple and clear, easy-to-understand-and-grasp features; second: the simplification of the model can be easily applied to many fields, for example, the relationship between variables in the function model and the correlation matrix representation between parameters. Third, by constructing mathematical models, data information can be combined with the actual situation, thus realizing the characteristics of high accuracy of visualization.

### 2.2. Mapping (Modeling)

The concept of mapping (PERT): it has the properties of fixed state, regular change, and uncertainty and satisfies the measurable characteristics; i.e., there is a certain number or correspondence between variables. When analyzing a mathematical model, it is important to understand the domain of definition and its properties [13]. For the problem we are studying, it can usually be seen as a constraint or a function to describe the existence of some connection between the state quantities; and when it comes to the actual situation that needs to calculate some specific values with definite integrals, the mapping (PERT) is used as one of the solutions, which is also an important prerequisite for the study of variables. For example, according to the mathematical function (3), the corresponding map can be drawn as shown in Figure 4.

(3) $$\begin{array}{c} y=\left\{\begin{array}{c} x^{2}-4x+4,\left(x\geq 2\right)\\ \frac{x}{2}-1,\left(x<2\right) \end{array}\right). \end{array}$$

### 2.3. Drawing

The drawing function can complete the process of converting any data into drawing data. As we all know, the principles and methods of adult computer graphics provide many rendering algorithms for display technology. Scan conversion includes hidden surface removal, light mode, shadow, transparency and shadow, texture mapping, and antialiasing technology. In general, the rendering method provided by the graphics computer can meet the needs of the rendering module in the display technology, so the research on the rendering function is not the main issue of the display technology. However, as mentioned earlier, in some new fields of display research, rendering technology can also become an important research technology, such as volume rendering technology.

Volume rendering technology is a relatively important research technology, and volume rendering technology is based on the image lighting model. The basic principle is a method based on optical diagrams. This method maps the three-dimensional data field into the basic modeling unit of the system with transparency and voxel characteristics. The system describes various light spots, colors, and other light characteristics passing through the volume data field under certain lighting conditions and uses this to represent the internal information of the data field.

In traditional visualization models, we simply describe the data, but it is not possible to visualize the problem itself. Therefore, in order to better represent the mathematical ideas and methods applied to real-life problem solving, firstly, a solid diagram can be drawn to realize the function of software technology analysis; secondly, it can be converted into images, text, and other forms in computer language and expressed to the user through the combination of graphics and text; finally, the model can be processed on the computer using visualization tools to get the final result.

According to the different rendering order, the volume rendering algorithm can be divided into the volume rendering algorithm in the order of the image space and the volume rendering algorithm in the order of the object space. There are also certain differences between the two. The volume rendering algorithm occupies the image space from each pixel on the screen and emits light according to the direction of the view. These rays pass through a three-dimensional data field, and the same sampling is performed on the rays to find the sampling point. These rays pass through a three-dimensional data field, and the same sampling is performed on the rays to find the sampling point. The volume rendering algorithm occupies the object space according to a specific projection area and projection direction. Starting from a three-dimensional data field, project all the frames onto an image plane in a certain order, calculate the contribution of each data point, and obtain the final image on the screen. The typical representative of this type of algorithm is the method of throwing snowballs.

The commonly used method in the volume rendering algorithm described in this article is the ray casting algorithm. The principle of the algorithm is to decompose complex nonsimple objects into several small units; these units are called “blocks,” that is, a basic unit. In the actual calculation, there are often some seemingly contradictory but interconnected units, and the relationship between these units is often very complex, so how to simplify the processing of these units has become one of the key issues in the visualization algorithm; the most common processing method is the local optimal solution method.

The main advantage of the ray casting method is that the use of gradients to change the boundary of the material can better reflect the normal direction of the surface of the object; using the phone model, specular reflection, diffuse reflection, and environment reflection can achieve better lighting effects, and the sampling step can be adjusted to reflect local details.

### 2.4. Showing

The visualization display module is a function in the visualization-based student domain statistics software to provide data processing and graphical presentation. The system consists of three main parts: (1) raw data acquisition; (2) calculation and analysis of results output; (3) attribute assignment and weighting coefficients for input variables and other operations [14].

First, all information available within the scope of the defined original element is extracted, and then this information is converted into subblocks that represent the name, nature, and type of the data object in the visual display module, as needed. The subblocks representing the names of the data objects can be converted directly into the information contained in the visual display module, or the information can be encoded and then represented in numerical or pictorial form by a computer or software for the original elements' characteristic property variables and other related relationships.

### 2.5. Application of Mathematical Models to Inputs and Outputs of Economic Variables

The application of mathematical models in economic modeling is very broad and complex, and it is mainly used in the calculation and analysis of macroeconomics between factors of production, between capital and labor, and in the field of microeconomics. It is particularly important to use mathematical modeling to solve practical problems in some special cases.

### 2.6. Mathematical Production Function Model

A production function is a mathematical description of the quantitative relationship between factor inputs, product output, and technological progress in a production process. The production function can be used to describe a company or industrial production process. When studying macroeconomic problems, the production process can also be described by considering the whole economic system as a whole enterprise. It is widely used in economic theory research, production modeling, technical progress measurement, production capacity analysis, and economic forecasting. Since 1928, when the production function was proposed by researchers, economists have paid great attention to the production function. Production function models include Cobb-Douglas production function, constant elasticity of substitution production function, variable elasticity of substitution production function, and transcendental logarithmic production function [15].

The most widely used production function is the Cobb-Douglas production function whose general form is shown in the following formula:

(4) $$\begin{array}{c} Y={\text{AK}}^{\alpha }L^{\beta }. \end{array}$$

In the formula, *Y* represents output, *K* and *L* represent the input of capital and labor, *A*, *α*, and *β* are parameters and *A* > 0, 0 < *a* < 1, 0 < *β* < 1. The Cobb-Douglas production function is generally called the C-D production function.

There are some improved forms of the Cobb-Douglas production function. One of them is the transcendental production function, whose form is shown in the following formula:

(5) $$\begin{array}{c} Y={\text{AK}}^{\alpha }L^{\beta }e^{\alpha^{\prime }L+\beta^{\prime }L},A>0,\alpha^{\prime },\beta^{\prime }\leq 0. \end{array}$$

If *α*′ and *β*′ are equal to zero, the formula is simplified to the Cobb-Douglas production function form. Take the logarithm as shown in the following formula:

(6) $$\begin{array}{c} \ln\;Y=\ln\;A+\alpha \;\ln\;L+\beta \;\ln\;K+\alpha^{\prime }L+\beta^{\prime }K. \end{array}$$

For this function, the marginal product may rise before it eventually falls. This function also allows output elasticity and substitution elasticity to vary with input changes.

The second improved form of the Cobb-Douglas production function is the Zellner-Revankar production function, whose form is shown in

(7) $$\begin{array}{c} {\text{Ye}}^{\text{cy}}={\text{AL}}^{\alpha }K^{\beta },c\geq 0. \end{array}$$

Here, if *c* = 0, it is simplified to the form of Cobb-Douglas production function. Take the logarithm as shown in

(8) $$\begin{array}{c} \ln\;Y+\text{cY}=\ln\;A+\alpha \;\ln\;L+\beta \;\ln\;K. \end{array}$$

The third improved form of the Cobb-Douglas production function is the Nervo-Linstad production function, whose form is shown in

(9) $$\begin{array}{c} Y^{1+c\;\ln\;Y}={\text{AL}}^{\alpha }K^{\beta },c\geq 0. \end{array}$$

Here, if *c* = 0, it is simplified to the form of Cobb-Douglas production function.

The fourth improved form of the Cobb-Douglas production function is the transcendental logarithmic production function, and its form is shown in

(10) $$\begin{array}{c} \ln\;Y=\ln\;A+\alpha \;\ln\;L+\beta \;\ln\;K+\gamma \;\ln\;L\;\ln\;K+\delta {\left(\ln\;L\right)}^{2}+\varepsilon {\left(\ln\;K\right)}^{2}. \end{array}$$

### 2.7. MCD Mathematical Production Function Model for Analysis of Economic Production Function

The production function is a mathematical description of the quantitative relationship between the input of production factors, product output, and technological progress in the production process. Production functions can be used to describe company or industrial production processes. When studying macroeconomic issues, the entire economic system can also be regarded as a whole enterprise to describe the production process. It is widely used in the fields of economic theory research, production model establishment, technological progress measurement, production capacity analysis, and economic forecasting. Since the production function was proposed by researchers in 1928, economists have paid great attention to the production function. Production function models include Cobb-Douglas production function, fixed substitution elastic production function, variable substitution elastic production function, and transcendental logarithmic production function.

Since its inception, the Cobb-Douglas production function has been widely studied and applied by many economists due to its excellent economic properties and easy solution. The quantitative economic model derived from the Cobb-Douglas production function has been widely used in economic theory and production practice research. With the deepening of production and technology research and development, one-sided shortcomings have gradually appeared. The academic circles have never stopped arguing about this, and research on improvements and revisions will continue [16].

First of all, some basic properties of the Cobb-Douglas production function are very related to the actual production process. If the output elasticity does not change, the factor substitution elasticity is 1. For the same research object, if the sampling interval is different, the output elasticity and factor substitution elasticity should be different. Although the research objects are the same and the sampling interval is the same, for different sample data points, because the ratio of input factors to production factors is different, the elasticity of output and the elasticity of substitution must be different.

Second, this model is limited in structure. The relationship and structure of variables in the economic system are very complex, which leads to the fact that the Cobb-Douglas production function often cannot match historical data with satisfactory accuracy in practical applications. Reason analysis shows that, with the advancement of science and technology, the innovation of production equipment, the improvement of production department functions, the improvement of production efficiency, and the diversification of products, the production process of most enterprises or industries shows the characteristics of multiple input elements and diversified structures. The entire production process of most enterprises or industries may have subproduction processes, and these subproduction processes are mutually influencing and interrelated. When scholars need to use the production function to describe the total production output of a specific company or industry and the functional relationship between capital and labor input, they often use indicators such as average production elasticity and average technological progress. It is not difficult to see from the form of the Cobb-Douglas production function that it is suitable for describing the input-output relationship that represents a single production process. It is difficult to describe the complex production structure using Cobb-Douglas production function. This requires people to develop new production functions.

In actual economic production activities, the entire production process of a company or industry with a diversified production structure consists of several subproduction units. Based on the previous discussion, coupled with the idea of additive nonparametric regression model, it is reasonable to assume that a production function showing this input-output relationship must be a combination of several basic production functions. That is, a model is a group of production subunits used to express each other's effects. Because the Cobb-Douglas production function has good economic properties, it is widely used by economists. This article assumes that a reasonable production function model should be a composite of several Cobb-Douglas production functions, expressed as

(11) $$\begin{array}{c} Y=F\left(K,L\right)=F\left(K^{\alpha_{1}}L^{\beta_{1}},K^{\alpha_{2}}L^{\beta_{2}},\ldots ,K^{\alpha_{m}}L^{\beta_{m}}\right). \end{array}$$

Therefore, this paper constructs a production function with the characteristics of multiple production structure, which is used to describe the input-output function relationship of a certain industry and enterprise. The specific form is shown in

(12) $$\begin{array}{c} Y=\sum_{i=1}^{m}A_{i}K^{\alpha_{i}}L^{\beta_{i}}. \end{array}$$

It is reversed from the digital form. This article calls this type of power exponential summation production function called MCD production function (Modified Cobb-Douglas Production Function). It can not only maintain some good properties of the Cobb-Douglas production function, but also improve the fitting accuracy of the production function to historical data. At the same time, it can also reflect the diversified structural characteristics of production to a certain extent [17].

The econometric form of the MCD production function is shown in

(13) $$\begin{array}{c} Y=\sum_{i=1}^{m}A_{i}K^{\alpha_{i}}L^{\beta_{i}}+\mu . \end{array}$$

In order to make the expression concise, suppose the Ai in the MCD production function is expressed as

(14) $$\begin{array}{c} A=\sum_{i=1}^{m}A_{i},\lambda_{i}=\frac{A_{i}}{A}. \end{array}$$

The above hypothetical model (11) can be expressed as shown in the following formula:

(15) $$\begin{array}{c} Y=A\sum_{i=1}^{m}\lambda_{i}K^{\alpha_{i}}L^{\beta_{i}}+\mu . \end{array}$$

## 3. Experimental Analysis and Results

### 3.1. Input-Output Line Model

Suppose that the economy of a country (or region) is divided into *n* sectors, and each sector produces one (or one type of) product, the total of intermediate use and final use in each department, minus transfers and imports. This result is equal to the total output of the department, as shown in

(16) $$\begin{array}{c} \sum_{j=1}^{n}x_{\text{ij}}+\left(r_{i}+p_{i}+q_{i}+c_{i}+s_{i}+d_{i}+e_{i}\right)-o_{i}-i_{i}=y_{i},i=1,2,\ldots ,n. \end{array}$$

Let *z*_*i*_=*r*_*i*_+*p*_*i*_+*q*_*i*_+*c*_*i*_+*s*_*i*_+*d*_*i*_+*e*_*i*_ − *o*_*i*_ − *i*_*i*_; get the following formula:

(17) $$\begin{array}{c} \sum_{j=1}^{n}x_{\text{ij}}+z_{i}=y_{i},\;i=1,2,\ldots ,n. \end{array}$$

The direct consumption coefficient is the core of the static input-output model. It can organically combine economic factors with technical factors, and it can combine technical factors for economic analysis. In a certain period of time, if the role of production technology and intermediate products does not change, it can be considered that aij is relatively stable. Substitute *x*_*ij*_ = *a*_*ij*_*x*_*ij*_ into formula (17) to obtain

(18) $$\begin{array}{c} \sum_{j=1}^{n}a_{\text{ij}}x_{j}+z_{i}=y_{i},\;i=1,2,\ldots ,n. \end{array}$$

### 3.2. Input-Output Column Model

The production input of each department is composed of three parts, namely, intermediate input, fixed asset depreciation, and initial input. From this, a balance equation can be obtained as shown in

(19) $$\begin{array}{c} \sum_{i=1}^{n}x_{\text{ij}}+E_{j}+w_{j}+b_{j}+t_{j}+m_{j}=x_{j},\;j=1,2,\ldots ,n. \end{array}$$

Marked as *h*_*j*_=*E*_*j*_+*w*_*j*_+*b*_*j*_+*t*_*j*_+*m*_*j*_, then formula (19) can be changed to

(20) $$\begin{array}{c} \sum_{i=1}^{n}x_{\text{ij}}+h_{j}=x_{j},\;j=1,2,\ldots ,n. \end{array}$$

Write the above formula in matrix form; get the following formula:

(21) $$\begin{array}{c} A_{c}X+H=X, \end{array}$$

where *H*=(*h*_1_, *h*_2_,…, *h*_*m*_)^*T*^ is the value-added column vector, as shown in

(22) $$\begin{array}{c} A_{c}=\left(\begin{array}{ccc} \overset{n}{\underset{i=1}{\sum }}a_{i1} & \; & \;\\ \; & \ddots & \;\\ \; & \; & \overset{\text{n}}{\underset{\text{i}=1}{\sum }}a_{\text{in}} \end{array}\right). \end{array}$$

### 3.3. Revision Method of the Input-Output Direct Consumption Coefficient

The direct consumption coefficient is the basis for calculating the absolute consumption coefficient and establishing the mathematical model. The accuracy of the consumption coefficient directly affects the overall balance and quality of the plan. In order to ensure the accuracy of the direct consumption coefficient, it is important to master the quality of basic statistical data. At the same time, it is necessary to understand some factors that directly affect consumption changes before the coefficient can be corrected.

In the revision of the visual model, the variables defined in the input-output model can be directly referenced, or they can be transformed into a correction independent of the established functions and not dependent on other known information. However, this approach is flawed in practical applications. If the previous year's data is used as the reference object, the estimation results will be biased from the real situation; if the time series factors are taken into account in the next year and the next months' statistics, we get a constant that was not included in the previous calculation of the variables defined in the visualization model and therefore cannot be revised directly, but only as a variable [18].

The establishment of the input-output model should follow the following principles:

1. The economic variables and GDP per capita are linearly related over a certain period of time, and their trends are basically consistent
2. There is interdependence between economic phenomena and other factors for a specific unit in the field under study

The following issues should be noted when constructing a mathematical visualization and quantitative analysis framework. Firstly, the relationship between quantitative and qualitative analysis should be paid attention to when constructing the mathematical visualization model. Secondly, the mathematical model should reflect the scientific and artistic aspects as much as possible. Finally, the indicators should be selected, adjusted, and applied according to the actual situation to meet the requirements of the prudence principle.

Today the direct consumption factor method has undergone many changes and it is mainly divided into nonmathematical methods and mathematical methods. Nonmathematical methods are such as the actual survey method and the expert assessment method. There is a mathematical method: the most basic one is the RAS method.

The RAS correction method is a direct consumption coefficient correction method, which is essentially an iterative correction method. The basic assumption of the RAS correction method is that the direct consumption coefficient changes come from two aspects.

The RAS method was proposed by the researcher Richard Stone in the 1960s. This method is also known as the bilateral proportional method. The idea of this method is to use the total average annual usage as the control amount for rows, and the average total input in the target year as the control amount for columns. The intermediate input matrix lists the conditions for double reduction, full utilization of the target year, and full input in the target year. Estimates are made using conventional statistical data, which greatly reduces the cost of the input-output table.

The most basic mathematical method in the direct consumption factor method is the RAS method, which has many advantages. (1) Using RAS directly as the basic idea of the correction model can make the calculation results more intuitive and clear, and it does not require any complicated and tedious mathematical steps in practical operation. (2) The visualization method enables us to observe, analyze, and understand the data from more perspectives.

## 4. Results

(1) The input-output model can be used to study many important proportional relationships in the national economy, which can be used to measure issues such as production or technological progress. For example, it can study the rate of intermediate products and the rate of final products, the value composition of products in a certain department, and so on.
(2) Study the impact of changes in each final demand on the output value of each department, labor remuneration, and social net income, for example, the increase and decrease of the military budget, the expansion and compression of the scale of infrastructure construction, and the impact of the increase and decrease of imports and exports on the national economy.
(3) Analyze the impact of changes in wages and taxes on the prices of products in each department. △*P*, △*V*, and △*M* are used to represent the column vectors composed of changes in prices, wages, and profits and taxes, respectively, as shown in
  (23) $$\begin{array}{c} \Delta P={\left(I-A^{T}\right)}^{-1}\Delta V,\Delta P={\left(I-A^{T}\right)}^{-1}\Delta M. \end{array}$$
(4) Analyze the impact of changes in the price of a product on the prices of other products.
(5) Conduct energy consumption analysis. Use the input-output table to calculate A and B, and further calculate the energy consumption indicators of the unit output value of the main sectors of the national economy. This is an important technical indicator, from which we can see the technical content and energy waste of products in the leading sectors of our national economy. It is helpful to find the gap and reduce the comprehensive energy consumption per unit of product.

## 5. Conclusions

In short, the application of scientific computing visualization technology can greatly accelerate data processing, and it can realize image communication between people and computers. It also enables scientists to guide and control the calculation process and consciously control scientific calculations so that they can run. The development of scientific computing visualization technology will further modernize scientific research equipment and the environment. It can thereby fundamentally change the diversity of scientific research, which has very important scientific significance. This paper focuses on the application of mathematical models based on scientific visualization in economic variables. The paper is divided into four major parts: theoretical part, algorithmic part, data processing part, and application part. The theoretical part mainly describes the theoretical knowledge related to scientific scientific visualization techniques, economic variables, mathematical models, etc. The algorithmic part mainly analyzes the mathematical production functions. The data processing part focuses on the use of scientific visualization techniques for economic data processing. The application part mainly describes the application of scientific visualization techniques in the analysis of economic variables and the application of mathematical model functions in the input and output models of economic variables. Through this study, we can learn that, in the process of economic development of enterprises, the level of technology, production efficiency, and capital costs have a certain influence on the direction and track of economic development, so enterprises should pay attention to various influencing factors in the process of development, so as to promote more “healthy” development of enterprises.

## Figures and Tables

**Figure 1:** Research model based on visual analysis.

**Figure 2:** Data preprocessing flowchart.

**Figure 3:** Flowchart of data compression technology.

**Figure 4:** Function map.

**Algorithm 1:** Processing of economic variable data.

## Data Availability

The data used to support the findings of this study are available from the corresponding author upon request.
